# Improving Arabic Sentiment Analysis Using CNN-Based Architectures and Text Preprocessing

**DOI:** 10.1155/2021/5538791

**Published:** 2021-09-06

**Authors:** Mustafa Mhamed, Richard Sutcliffe, Xia Sun, Jun Feng, Eiad Almekhlafi, Ephrem Afele Retta

**Affiliations:** School of Information Science and Technology, Northwest University China, Xi'an, China

## Abstract

Sentiment analysis is an essential process which is important to many natural language applications. In this paper, we apply two models for Arabic sentiment analysis to the ASTD and ATDFS datasets, in both 2-class and multiclass forms. Model MC1 is a 2-layer CNN with global average pooling, followed by a dense layer. MC2 is a 2-layer CNN with max pooling, followed by a BiGRU and a dense layer. On the difficult ASTD 4-class task, we achieve 73.17%, compared to 65.58% reported by Attia et al., 2018. For the easier 2-class task, we achieve 90.06% with MC1 compared to 85.58% reported by Kwaik et al., 2019. We carry out experiments on various data splits, to match those used by other researchers. We also pay close attention to Arabic preprocessing and include novel steps not reported in other works. In an ablation study, we investigate the effect of two steps in particular, the processing of emoticons and the use of a custom stoplist. On the 4-class task, these can make a difference of up to 4.27% and 5.48%, respectively. On the 2-class task, the maximum improvements are 2.95% and 3.87%.

## 1. Introduction

Users of social media platforms like Facebook, Twitter, and Instagram display a huge number of personal emotions and attitudes. For example, they may complain about the product they have purchased, discuss current issues, or express their political views. The use of information obtained from social media is key to the operation of many applications such as recommendation systems, organizational survey analyses, or political campaign planning [1]. It is very important for governments to analyze public opinion because it explains human behavior and how that behavior is in turn influenced by the opinions of others. The inference of user sentiment can also be very useful in the area of recommender systems and personalization to compensate for the lack of explicit user feedback on a provided service.

There are many languages used on the Internet. According to [2], Arabic is ranked 4th in the world, with 237 million Internet users. Therefore, it is important to develop sentiment analysis tools for this language. Arabic is the most active member of the community of Semitic languages in terms of speakers, being used in North Africa, the Middle East, and the Horn of Africa. It has three classes, modern standard Arabic (MSA), dialect Arabic (DA), and classical Arabic (CA) [3]. MSA is used in formal contexts, such as news reporting, schools, and marketing forums. By contrast, in informal writing, particularly in social media, Arabic dialects are used and differ from country to country. Classical Arabic is used in religious scriptures such as the Holy Qur'an and for prayer. While automatic sentiment analysis (SA) is an established subject of study, it is well known that there are many challenges specifically related to Arabic [4]:

- Words are connected to each other, making tokenization difficult.
- Both words and sentences in Arabic can be very long.
- A word can have many meanings in Arabic. For example, some names in Arabic originate from adjectives; while the adjective may express a positive or negative sentiment, the name itself does not. For example, the name “Jameelah” and the adjective pretty are both written as in Table 1.
- Different users can write the same word in different directions, for example, see Ta'marbootah in Table 1.
- Based on whether the subject of a verb is singular or plural, that verb may be written in various forms.
- The same applies to male or female, for instance, “He likes cars” and “She likes cars” in Table 1.  Idioms may be used by Arabic speakers to express their thoughts, and an expression may possess a tacit thought. For instance, the last example in Table 1 expresses a negative opinion even though there is no negative word in it.

Below are the main contributions of this work:

- We propose models MC1 and MC2 for Arabic sentiment analysis, for both 2-way and n-way classifications. MC1 is a convolutional neural network (CNN) with an average-max-pooling function with two layers; it is capable of using different lengths and weights of windows for the number of feature maps to be created.
- Model MC2 is a CNN using bidirectional gated recurrent units (GRUs).
- We pay close attention to Arabic preprocessing issues such as tokenization, strip elongation, normalization, and stopword design.
- The classification performance of our methods exceeds current baselines for Arabic.
- We demonstrate by an ablation study that our novel preprocessing steps contribute to the superior performance.
- Our methods work with high efficiency; thus, they can be applied to very large datasets.

The paper is organized as follows.  Section 2 reviews previous work on Arabic sentiment analysis using deep learning.  Section 3 describes the proposed architectures and processing methods.  Section 4 presents our experiments.  Section 5 gives conclusions and suggests future work.

## 2. Previous Work

Sentiment analysis has been carried out using many machine learning and deep learning approaches and in many different languages (Table 2). We will first start with non-Arabic sentiment analysis and later focus on Arabic.  Table 3 summarises some of the previous work on non-Arabic sentiment, showing the dataset, model, and result reported. However, this has become a very active area and the main focus of this paper is on Arabic. For comprehensive recent surveys dealing with work in other languages, see Dang et al. [35] and Oueslati et al. [1].

Kim [10] applied convolutional neural networks (CNNs), working over word vectors, to several language processing tasks, including sentiment analysis. This showed the potential of such an approach. Zhou et al. [17] adopted a form of CNN where the dense layer is replaced with a long short-term memory (LSTM) layer. The output of the convolution is fed to the LSTM layer thus combining the benefits of each process. The method was applied to sentiment classification with the Stanford Sentiment Treebank (SST) dataset [36].

Onan et al. [37] used three association rule mining algorithms, Apriori, Predictive Apriori, and Tertius on educational data. Predictive Apriori was the most effective (99%). Onan et al. [21] also utilized machine learning, ensemble methods, and latent Dirichlet allocation (LDA) on four sentiment datasets [38]. The machine learning methods were Naive Bayes (NB), support vector machines (SVMs), logistic regression (LR), radial basis function networks, and K-nearest neighbour (KNN). Ensemble methods included bagging, AdaBoost, random subspace, voting, and stacking. An ensemble with LDA gave the highest accuracy (93.03%). Onan et al. [39] further implemented statistical keyword extraction methods on an Association for Computing Machinery document collection for text classification. Using the most frequent keywords along with a bagging ensemble and random forests gave the highest accuracy. Finally, Onan [40] used NB, SVMs, LR, and the C4.5 decision-tree classifier to perform a number of text classification tasks. Ensemble methods included AdaBoost, random subspace, and LDA. The eleven datasets were taken from Rossi et al. [38]. Combining a cuckoo search algorithm and supervised K-Means gave an accuracy of 97.92%.

Paredes-Valverde et al. [11] used a CNN with Word2vec, SVM, and NB on their own Spanish Sentiment Tweets Corpus. The CNN model gave a better performance than traditional methods (88.7%).

Chen et al. [5] used an adversarial deep averaging network (ADAN) model [41] to transfer the knowledge learned from labeled data on a resource-rich source language to a low-resource language where only unlabeled data exist. They used the Arabic Sentiment Tweets Dataset (ASTD) [28] and the MioChnCorp Chinese dataset [42] (with accuracies of 54.54% and 42.49%, respectively).

Attia et al. [9] applied a CNN to three datasets, one each in English, German, and Arabic. These were the Sanders Twitter Sentiment Corpus (STSC) [43], the German Germeval Dataset (GGD) [44], and ASTD. The best Arabic result was 67.93% using oversampling.

Onan [20] focused on the five Linguistic Inquiry and Word Count (LIWC) categories and used their own corpus of Twitter tweets. He applied NB, SVMs, LR, and KNN classifiers, as well as three ensemble learning methods, AdaBoost, bagging, and random subspace. The most successful approach (89.1%) was to combine linguistic processes, psychological processes, and personal concerns with the NB random subspace ensemble. Onan [45] carried out an extensive comparative analysis of different feature engineering schemes with machine learning and ensemble methods for text genre classification. This further showed the potential of such methods for identifying sentiment.

Li et al. [16] applied CNN-LSTM and CNN-BiLSTM models incorporating Word2vec and GloVe embeddings to two datasets, Stanford Sentiment Treebank (SST) [36] and a private Chinese tourism review dataset. They adopted a novel padding method compared with zero paddings and showed that it improves the performance. The best model was CNN-LSTM with 50.7% (SST) and 95.0% (Chinese) accuracies.

Onan [23] used machine learning and deep learning on a balanced corpus containing student evaluations of instructors, collected from ratemyprofessors.com. The recurrent neural network (RNN) with attention and GloVe embeddings gave the highest accuracy (98.29%). Onan [24] applied machine learning, ensemble learning, and deep learning methods to a balanced corpus of massive open online courses (MOOCs). Similar to Onan [23], an RNN combined with GloVe gave the best performance (95.80%). Onan and Toçoğlu [46] once again focused on MOOC discussion forum posts, working with a 3-way text classification model. There were three stages of processing, word-embedding schemes, weighting functions, and finally clustering using LDA. The best accuracy was attained by a Doc2vec model with a term frequency-inverse document frequency (TF-IDF) weighted mean and divisive analysis clustering. Finally, Onan and Toçoğlu [6] utilized a three-layer stacked BiLSTM with Word2vec, FastText, and GloVe. The task was sentiment classification using three sarcasm datasets, one collected by themselves, the second based on the Internet Argument Corpus [47], and finally the News Headlines Dataset for Sarcasm Detection [48]. Two weighting functions and eight supervised term weighting functions were tried. A trigram-based configuration with inverse gravity moment-based weighting and maximum pooling aggregation was the fastest and best performing (95.30%).

Behera et al. [15] proposed a Co-LSTM model combining CNN and LSTM; there were four datasets, IMDB [49], Airline Reviews [50], Self-Driving Car [51], and US Presidential Election [49]. The results were 83.13%, 94.96%, 86.43%, and 90.45%, respectively.

We will now summarise the architectures used in the above works to analyze sentiment in non-Arabic documents. Paredes-Valverde et al. [11] and Behera et al. [15] used machine learning models such as NB, RF, and SVM. On the other hand, Onan et al. [20, 21] utilized ensemble machine learning models. Paredes-Valverde et al. [11] also applied CNN, Behera et al. [15] used Co-CNN, and Li et al. [16] used CNN-LSTM and CNN-BiLSTM. Finally, Onan et al. [6, 23, 24] applied RNN, LSTM, and Bi-LSTM.

Next, we will focus our review on approaches to sentiment analysis applied to the Arabic language.  Table 4 summarises recent work, showing the dataset, split, model, and result reported. Baly et al. [25] used two approaches, machine learning and deep learning. Three models were based on support vector machines (SVMs): Baseline, All Words, and All Lemmas. Two further models used recursive neural tensor networks (RNTNs): RNTN Words and RNTN Lemmas. Evaluation was against the Arabic Sentiment Tweets Dataset (ASTD) [28]. The best results were accuracy = 58.5% and average F1 = 53.6% for the RNTN Lemmas model.

Heikal et al. [13] used CNN, LSTM, and ensemble models against the ASTD. For the ensemble model, accuracy was 65.05%. Their methods show a better result than that of the RNTN Lemmas model [25].

Lulu and Elnagar [7] used LSTM, CNN, BiLSTM, and CNN-LSTM. Training was performed with texts in three Arabic dialects, using the Arabic Online Commentary (AOC) dataset [27]. The corresponding subset is composed of 33K sentences equally divided between Egyptian (EGP), Gulf including Iraqi (GLF), and Levantine (LEV) dialects. Results show that LSTM attained the highest accuracy with a score of 71.4%.

Alnawas and Arici [19] used a word embedding model, logistic regression, decision trees, support vector machines (SVMs) [52], and Naive Bayes. The training data were the Iraqi Arabic Dialect (IAD) [31]. The best result was *P* = 82%, *R* = 79%, and *F*1 = 78%.

Dahou et al. [18] applied DE-CNN to five datasets: ArTwitter [53], STD [30], AAQ, ASTD-2 [28], and AJGT [54]. AAQ consisted of more than 4000 tweets extracted from ASTD, ArTwitter, and QRCI . Arabic word embeddings for the model were taken from Altowayan and Tao [55]. The DE-CNN model gave accuracies of 93.44%, 75.33%, 87.16%, 81.54%, and 92.81% on these datasets, respectively.

Soufan [14] applied Multinomial Naive Bayes (MNB), SVM [52], LSTM, and CNN [56] to both a binary dataset and a multiclass dataset. For SemEval [33], the CNN-Word [12] model achieved 50.1% accuracy, the highest in the SemEval task. For the binary classification, the machine learning models achieve better accuracy than the other models.

Kwaik et al. [22] used an LSTM Baseline [57], a Kaggle Baseline, and their LSTM-CNN model with three datasets: Shami-Senti [34], Large-Scale Arabic Book Review (LABR) [32], and ASTD. In two-way classification, the LSTM-CNN model attained accuracy of 93.5% (Shami-Senti) and 85.58% (ASTD). In three-way classification, results are 76.4% (Shami-Senti), 66.4% (LABR 3), and 68.6% (ASTD).

We now summarise the architectures used in the above works to analyze sentiment in Arabic documents. Baly et al. [25] used an approach based on binary parse trees with compositional combination of constituent representations, followed by a softmax classifier. Alnawas and Arici [19], Soufan [14], and Kwaik and Chatzikyriakidis [26] used machine learning models. Dahou et al. [18] proposed the DE-CNN model, a CNN exploiting the ability of the DE algorithm. Chen et al. [5] used an ADAN to transfer knowledge from one language to another. Attia et al. [9] used a model based on CNN while Lulu and Elnagar [7] used LSTM. Heikal et al. [13] and Kwaik et al. [22] combined CNN with LSTM. Our two proposed approaches are based on CNN and CNN through BiGRU, respectively (see next section).

Finally, we are particularly interested in the use of emojis (small images such as the smiley face) and emoticons (similar images constructed from keyboard characters, e.g., 8)). Al-Twairesh et al. [58] have used emojis to extract tweets which might contain emotional content. Kwaik et al. [26] also used emojis for this purpose and within an iterative algorithm for classifying a large dataset. Baly et al. [25] extracted both emoticons and emojis and replaced them with special tokens which are input to the training process along with the text. We use similar methods and measure the exact effect of emoticons on training.

## 3. Proposed Method

### 3.1. Outline

We apply our text cleaning and preparation methods to address the challenges of Arabic tweets. For tokenization, we used the Natural Language Toolkit (NLTK), and then we applied methods MC1 and MC2 working with both multiclass classification and binary classification. We trained and tested on the ASTD Arabic dataset [28] and also the larger ATDFS dataset [59].

### 3.2. Text Preprocessing and Normalization Steps

Our approach focuses in particular on preprocessing because this is a key aspect of Arabic text analysis, as discussed above.  Table 5 shows 22 preprocessing steps which have been used for Arabic, while Table 6 shows the exact steps used by recent papers. On the bottom line of the table are the steps used in the proposed approach.

Steps 1 and 2 are concerned with the removal of Twitter-specific metadata, for example, that shown in this JSON sample of metadata:

  “User”: {
  “id”: 6253282,
  “id_str”: “6253282”,
  “name”: “Twitter API”,
  “location”: “Saudi Arabia, Riyadh”
  }

Step 3 removes digits from texts, including dates. Steps 4 and 5 deal with repeated characters in Arabic words. This is derived from Kwaik et al. [34] and used in Kwaik et al. [22]. Step 6 removes characters such as ‘÷×_-“...”!|+,´.?:¨/][%&̂^*∗*^()<>;. Step 7 removes punctuation. Step 8 removes diacritics like fatha, damma, kasra, tanween fatha, tanween damma, tanween kasra, shadda, and sukuun. Diacritics are very important in Arabic to determine the correct pronunciation, but for text processing, they can be removed. Step 9 deletes any non-Arabic text such as English or French words. The aim is to standardise the text. Step 10 removes emojis, which are small digital images expressing emotion. Step 11 eliminates duplicated tweets as they do not add further information. Step 12 corrects elongated words and carries out other Arabic normalization steps (see Table 7). Elongation in Arabic is connected with the pronunciation of a word, not its meaning. So, this step helps to reduce text size and improve word recognition, assisting in identifying and controlling word length. Step 13 replaces an emoticon like (: with its meaning (Table 8). Step 14 combines the removal of hashtags “#” with the removal of word elongations. Step 15 removes comment symbols such as the heart symbol, dove symbol, raven symbol, tree symbol, and owl symbol. Steps 16 and 17 are concerned with the choice of tokenizer. Some Arabic words contain stopwords such as substrings, and tokenization can separate them. Also, there are some symbols and characters which are part of a word, but on tokenizing, the word will be wrongly divided into parts. For high accuracy in sentiment classification, it is important for the tokenizer to handle these cases correctly. Step 18 is manual tokenization, only used by Attia et al. [9]. Steps 19 and 20 specify the choice of stoplist. The NLTK Arabic stoplist (step 19) contains 248 words; we increase the vocabulary for our stoplist to 404 words, 2,451 characters in total. We create additional stopwords because users of social media are not only writing modern standard Arabic but also using dialects. So, our additional stopwords (see Table 9) help to remove noise and improve the results. Steps 20 and 21 are concerned with document and line processing and are only used in Alnawas and Arici [19].

In conclusion, steps 15, 17, 19, and 20 are unique to the proposed approach. Moreover, our preprocessing is much more comprehensive than that in previous works, as Table 5 shows.

### 3.3. Text Encoding

#### 3.3.1. Input Layer

In order to start, let us assume that the input layer receives text data as *X*(*x*_1_, *x*_2_,…, *x*_*n*_), where *x*_1_, *x*_2_,…, *x*_*n*_ is the number of words with the dimension of each input term *m*. Each word vector would then be defined as the dimensional space of *R*^*m*^. Therefore, ℝ^*m*×*n*^ will be the input text dimension vacuum.

#### 3.3.2. Word Embedding Layer

Let us say the vocabulary size is *d* for a text representation in order to carry out word embedding. Thus, it will represent the dimensional term embedding matrix as *A*^*m*×*d*^. The input text *X*(*x*_*I*_), where *I* = 1,2,3,…, *n*, *X* *ϵ* ℝ^*m*×*n*^, is now moved from the input layer to the embedding layer to produce the term embedding vector for the text. Word representations for modern standard Arabic (MSA) were implemented using the AraVec [60] word embedding pretrained by Word2vec [61] on Twitter text. The representation of input text *X*(*x*_1_, *x*_2_,…, *x*_*n*_)*ε*ℝ^*m*×*n*^ as numerical word vectors is then fed into the model. *x*_1_, *x*_2_,…, *x*_*n*_ is the number of word vectors with each dimension space *R*^*m*^ in the embedding vocabulary.

### 3.4. Proposed Two Architectures for Arabic Sentiment Analysis

We use two network architectures in this work. First, MC1 is a convolutional neural network (CNN) with global average pooling function with two layers; it is capable of using different lengths and weights of windows for the number of feature maps to be created and can be used for both dual and multiple classifications. Second, MC2 is a CNN using bidirectional gated recurrent units (GRUs). The CNN with a max-pooling function can process our inputs in two directions, forward and backward. As is well known, this solves long sequence training issues and can improve efficiency and accuracy.

MC1 (Figure 1) consists of embedding layers containing max-features = num-unique-word (which varies for each dataset), embedding-size = 128, and max-len set to {150,50,30}; after that there is a convolutional neural network layer with 512 filters, having kernel size = 3, padding = “valid,” activation = ReLU, and strides = 1. There is then a global average pooling 1D, with pool size = 2, followed by another convolution layer with 256 filters, having kernel size = 3, padding = “valid,” activation = ReLU, and strides = 1. We apply the regularization technique on the previous layer, having 256 filters and the ReLU activation function. This helps us to reduce model capacity while maintaining accuracy. Next, there is batch normalization, and finally a fully-connected softmax layer, to predict the output from four sentiment classes: positive, negative, neutral, and objective.

MC2 (Figure 2) consists of embedding layers containing max-features = num-unique-word (which varies for each dataset), embedding-size = 128, and max-len set to {150,50,30}; after that there is a convolutional neural network layer with 128 filters, having kernel size = 3, padding = “valid,” activation = ReLU, and strides = 1. There is then a maxpooling 1D, with pool size = 2, followed by another convolutional neural network layer with 64 filters, having kernel size = 3, padding = “valid,” activation = ReLU, and strides = 1. This is followed by a maxpooling 1D having pool size = 2, and then a dropout = 0.25. There is next a SpatialDropout1D = 0.25 for the bidirectional gated recurrent unit layer consisting of 128 units, then a dropout = 0.5, then a flattened layer followed by a dense layer of 128 units, and activation = ReLU. After that there is a dropout = 0.5, and finally a fully connected softmax layer to predict the sentiment class.

## 4. Experiments

### 4.1. Datasets

For sentiment classification of Arabic text, our models are trained using the Arabic Sentiment Tweets Dataset (ASTD) [8, 28] and the Arabic Twitter Data For Sentiment (ATDFS) [29, 59]. Tables 10 and 11 show the details of the datasets.

ASTD contains versions in two, three, and four emotion classes. ASTD (4C) consists of 10,006 Arabic tweets, with 4 classes (799 subjective positive tweets, 1,684 subjective negative tweets, 832 subjective mixed tweets, and 6,691 objective tweets) [28]. ASTD (3C) consists of three classes, 665 positive tweets, 1,496 negative tweets, and 738 neutral tweets. ASTD (2C) consists of two classes, 799 positive tweets and 1,684 negative tweets. ATDFS [59] consists of two classes, 93,144 positive tweets and 63,263 negative tweets.

### 4.2. Experimental Settings

We used our own tuning and hyperparameter values. The settings for the experiments are shown in Table 12. We used the TensorFlow framework for the implementation (the source code for this paper is available at https://github.com/mustafa20999/Improving-Arabic-Sentiment-Analysis-Using-CNN-Based-Architectures-and-Text-Preprocessing).

### 4.3. Experiment 1: Multiclass Sentiment Classification

In the first stage, the proposed models MC1 and MC2 were applied to the multiclass version of ASTD. First, the data were split into 80/10/10 train/validation/test. Second, the data were split 70/10/20 to allow direct comparison with Baly et al. [25] and Heikal et al. [13].

In the second stage, an ablation study was carried out to establish the effect on performance of the preprocessing. First, step 13 was removed from the preprocessing and the training was repeated. Second, step 13 was replaced and step 20 was removed and training was repeated.

In each case, we used 10-fold cross validation and reported the average result.

### 4.4. Experiment 1 Results

Results are presented in Table 13. For each task, we provide the best previous result as a baseline. For 4-class task and the 80/10/10 split, MC2 achieves 73.17% accuracy, compared to the baseline of 65.58% [29]. For 4-class task and the 70/10/20 split, MC2 achieves 70.23% compared to the baseline of 65.05% [13]. On 3-class, MC2 achieves 78.62% compared to the baseline of 68.60% [22]. Concerning the ablation study, we must compare Table 13 with Tables 14 (step 13 removed) and 15 (step 20 removed). Recall that step 13 is the replacement of emoticons with their equivalent meaning, and step 20 is the use of a custom stoplist (Tables 8 and 9).

For the removal of step 13 (Table 14), we can see that the best results for ASTD (4C, 80/10/10) and ASTD (3C, 80/10/10) (73.17%, 78.62%) are reducing to (70.32%, 74.35%), changes of −2.85% and −4.27%, respectively. So, simply giving meaning to emoticons is resulting in an improvement of several percent for the 80/10/10 splits. It would be interesting to investigate whether the effect of emoticons on prediction varies across the different emotion classes.

For the removal of step 20 (Table 15), the new figures are 68.38% and 73.14% and the changes are −4.79% and −5.48%. Here we see a larger change than that for the emoticons, just on the basis of the stoplist. So, the ablation study is supporting the hypothesis that preprocessing can make a significant difference to Arabic sentiment analysis, at least on social media tweets.

### 4.5. Experiment 2: Binary Sentiment Classification

The proposed models MC1-2 were applied to 2-class ASTD and 2-class ATDFS. In the second stage, the same ablation study was repeated, first removing Step 13 and then replacing step 13 and removing step 20. We used 10-fold cross validation and reported the average result.

### 4.6. Experiment 2 Results

Results are presented in Table 16 and all are 2-class. As before, we provide the best previous result as a baseline. For ASTD, MC1 achieves 90.06% accuracy (baseline 85.58% on 80/10/10 split [22]), while for ATDFS, MC2 achieves 92.96% accuracy (ATSAD baseline 86.00% [26]). The latter figure is from a similar dataset described in Kwaik and Chatzikyriakidis [26], as we did not find a published baseline for ATDFS. For the ablation study, we compare Table 16 with Tables 17 (step 13 removed) and 18 (step 20 removed). For the removal of step 13, the new figure for ASTD and MC1 is 87.11%, a change of −2.95%. For the removal of step 20, the new figure is 86.19%, a change of −3.87%. For ATDFS, the new figures for MC2 are 90.86%, a change of −2.1%, and 89.68%, a change of −3.28%. These figures confirm the trends shown for the multiclass results.

### 4.7. Accuracy during Training

Figure 3 shows the validation accuracy of models MC1 and MC2 with the ASTD (4C) dataset after 50 epochs, with different splits.  Figure 4 shows accuracy against training epoch for MC1 and the ASTD dataset.

Figures 5 and 6 show the models' training and validation accuracy with the ATDFS dataset. At epoch 10, it shows us the different performances and also different times for predictions; for the MC2 model, elapsed time is 8 h33 m58 s (8 hours, 33 minutes, and 58 seconds) and for MC1, it is 2 h27 m17 s. Thus, MC1 gives us the best validation accuracy and least execution time.

## 5. Conclusion and Future Work

In this paper, we explained a comprehensive approach to Arabic text preprocessing before presenting two architectures for sentiment analysis using 2-class, 3-class, and 4-class classifications. Our results exceed current baselines. In an ablation study, we showed that the replacement of emoticons by content words and the use of a custom stoplist can each alter performance by several percent. This indicates that text preprocessing is very important for Arabic sentiment analysis.

In future work, we plan to look at the effect of preprocessing across sentiment categories and to apply sentiment analysis to more specific Arabic contexts.

## Figures and Tables

**Figure 1:** MC1 model architecture.

**Figure 2:** MC2 model architecture.

**Figure 3:** Accuracy during training for the 4-class ASTD. (a) Performance with ASTD (4C, 80 + 10+10); MC2 achieves the highest accuracy, 73.17%. (b) Performance with ASTD (4C, 70 + 10+20); MC2 achieves the highest accuracy, 70.23%. (c) For ASTD (3C), MC2 achieves the highest accuracy, 78.62%.

**Figure 4:** MC1 model accuracy with ASTD (2C).

**Figure 5:** MC1 model accuracy with ATDFS (2C).

**Figure 6:** MC2 model accuracy with ATDFS (2C).

**Table 1:** Arabic language challenges.

Arabic text	الصداقة تزرع الحياة أزهارًا
	Blossom life cultivates friendship

Names in Arabic originate from adjectives	جَمِيلةَ
	Incantations

Ta'marbootah, diverse directions	االمؤثره,االمؤثرة
	The influencer, the influential

Male or female	هو يحب السيارات , هي تحب السيارات
	He likes cars, she likes cars

Sentence has negative sentiment though there is no negative word in it	مسائل قدرات مهمة جدا وصعبة
	Capacity issues are very important and difficult

**Table 2:** Summary of sentiment analysis approaches (O = other languages, A = Arabic language, ADAN = adversarial deep averaging network, Bi-LSTM = bidirectional long short-term memory network, CNN = convolutional neural network, DT = decision tree, DE = differential evolution, LR = logistic regression, KNN = K-nearest neighbour, LDA = latent Dirichlet allocation, LSTM = long short-term memory, MNB = Multinomial Naive Bayes, NB = Naive Bayes, RNN = recurrent neural network, RNTN = recursive neural tensor network, and SVM = support vector machine).

Approach	Used in
ADAN	O: [5]
BiLSTM	O: [6]; A: [7]
CNN	O: [9–11]; A: [7, 12–14]
CNN-LSTM	O: [15–17]; A: [7]
CNN-BiLSTM	O: [16]
DE-CNN	A: [18]
DT	A: [19]
Ensemble	O: [20, 21]; A: [13]
KNN	O: [20, 21]
LDA	O: [21]
LR	O: [20, 21]; A: [19]
LSTM	A: [7, 13, 14, 22]
LSTM-CNN	A: [22]
NB/MNB	O: [11, 20, 21]; A: [14, 19]
RNN	O: [23, 24]
RNTN	A: [25]
SVM	O: [11, 20, 21]; A: [14, 19, 25, 26]

**Table 3:** Previous work on non-Arabic sentiment analysis.

Paper	Dataset	Split	Model	Result (%)
[10]	SST-2 (2C)	80 + 20	CNN	88.1
[17]	SST-1 (2C)	70 + 10 + 20	CNN-LSTM	87.8
[21]	Reviews (2C)	90 + 10	LDA	93.03
[11]	Spanish sentiment tweets (2C)	80 + 20	CNN	88.07
[9]	Sanders (4C)	80 + 20	CNN	78.3
[5]	MioChnCorp Chinese (5C)	80 + 20	ADAN	54.54
[20]	Twitter (3C)	70 + 30	Ensemble	89.10
[23]	Ratemyprofessors (2C)	90 + 10	RNN-AM	98.29
[16]	Chinese tourism reviews (2C)	90 + 10	CNN-LSTM	95.01
[24]	MOOC evaluations (2C)	80 + 20	GloVe + LSTM	95.80
[15]	Airline reviews (2C)	70 + 30	Co-LSTM	94.96
[6]	Sarcasm Corpus (2C)	80 + 20	Bi-LSTM	95.30

**Table 4:** Previous work on Arabic sentiment analysis.

Paper	Dataset	Split	Model	Result (%)
[25]	ASTD (4C)	70 + 10 + 20	RNTN lemmas	58.50
[5]	ASTD (4C)	50 + 50	ADAN	54.54
[9]	ASTD (4C)	80 + 20	CNN	67.93
[13]	ASTD (4C)	70 + 10+20	Ensemble	65.05
[7]	AOC (2C)	80 + 10+10	LSTM	71.40
[19]	IAD (2C)	80 + 20	SVM	78.00
[18]	ASTD (2C)	80 + 20	DE-CNN	81.89
[14]	ASTD (2C)	90 + 10	SVM	80.50
[22]	ASTD (3C)	80 + 10 + 10	LSTM-CNN	68.60
[22]	ASTD (2C)	80 + 10 + 10	LSTM-CNN	85.58
[26]	ATSAD (2C)	95 + 5	Complex model	86.00

**Table 5:** Preprocessing steps for Arabic sentiment analysis.

Num	Step
1	Remove Twitter API metadata: time and tweet ID
2	Remove location, username, and RTT
3	Remove all digits including dates
4	Remove all repeated characters
5	Remove all repeated characters by using algorithm
6	Remove special characters
7	Remove punctuation marks
8	Remove all diacritics
9	Remove non-Arabic characters
10	Remove emojis
11	Remove duplicated tweets and links
12	Correct elongated words
13	Replace emoticon with its equivalent meaning
14	Normalize hashtag “#” symbols, underscores in composite hashtags, and word elongations (letter repetitions)
15	Remove symbols such as owl, tree, and so on
16	Tokenize with Stanford CoreNLP
17	Tokenize with NLTK
18	Manually tokenize, inserting space between words and punctuation marks
19	Use NLTK stoplist
20	Use custom stoplist
21	Split document to a single line and split each line to a single word
22	Collect words for source line, collect lines for source documents, and clean comments

**Table 6:** Preprocessing steps in proposed method vs. previous work.

Paper	Preprocessing description
[25]	1, 4, 12, 13, 14
[5]	16
[9]	1, 2, 3, 7, 8, 18
[13]	1, 3, 4, 6, 7, 9
[7]	6, 7, 8
[19]	6, 7, 9, 14.21, 22
[14]	1, 3, 4, 7, 8, 9, 10, 11
[22]	3, 4, 5, 6, 7, 8, 9
[26]	1, 2, 3, 4, 6, 7, 8, 9, 13
Proposed method	1, 2, 3, 4, 6, 7, 8, 9, 11, 12, 13, 15, 17, 19, 20

**Table 7:** Text normalization rules.

Strip Elongation	موهوب ⟶ مــــــوهــــــوب
Normalize Hamza	ء ⟶ ى,ؤ
Normalize Alef	أ ⟶ ا,إ,ا
Normalize Yeh	ي ⟶ ى
Normalize Heh	ه ⟶ ة
Normalize Caf	ک ⟶ ك

**Table 8:** Examples of words and corresponding emoticons in Arabic.

Word	Emoticon
مرتبك وجهه	o.o
سعيد	(:
جدآ سعيد وجهه	∧_∧
غاضب وجهه	):<
بكاء	)':
شيطاني	(:3
ملائكي	O:)

**Table 9:** Examples from the custom stoplist.

أصلا,أصبح,أسكن
أمسي,أمس,أمد
تعلمّ,تعسآ,تشرين,تسعين,تحول تفعلون,تفعلان
جنية,جميع
صبرا, صراحة, صدقا, صبرا, صبر, صباح
طاق, طالما, طرا
مابرم, مادام, مارس, مافتئ, مازال
مساء,مرّة,مثل

**Table 10:** Arabic datasets for sentiment analysis.

Datasets	Language	Source	Size	#Classes	Balanced
AOC [27]	MSA + DIA	Twitter, Facebook, and news	110 K	3	N
ASTD [28]	MSA + DIA	Twitter	10 K	4	N
ATDFS [29]	MSA	Twitter	21.42 MB	2	N
ATSAD [26]	MSA + DIA	Twitter	36 K	2	Y
BBNASAD [30]	DIA	BBN posts	1.2 K	3	Y
IAD [31]	DIA	Facebook, news, and companies	250.2 K	2	Y
LABR [32]	MSA	Books	63 K	2, 3	N
SemEval [33]	MSA + DIA	Twitter	70 K	2	Y
Shami-Senti [34]	DIA	Twitter	2.5 K	3	N

**Table 11:** Datasets for our experiments.

Datasets	Positive tweets	Negative tweets	Mixed tweets	Irrelevant tweets	Neutral tweets	Total
ASTD (4C)	799	1,684	832	6,691	—	10,006
ASTD (3C)	665	1,496	—	—	738	2,899
ASTD (2C)	799	1,684	—	—	—	2,483
ATDFS (2C)	93,144	63,263	—	—	—	156,407

**Table 12:** Experimental settings.

Setting	Value (s)
Embedding size	{100, **128**, 200, **300**}
Pooling	{**2**, **4**, **6**, 8, 16}
Batch size	{**64**, **128**, **164**, **200**, 400}
Kernel size	{**3**, **5**, 7, 10}
Number-classes	{**2**, **3**, **4**, 5, 10}
Epoch	{5, **10**, 20, **50**, **100**, 200}
Optimizer	Adam
Learning rate	{0.01, **0.001**, 0.0001}

**Table 13:** Accuracy with multiclass ASTD datasets.

Models	Accuracy (%)		
	ASTD (4C, 80 + 10 + 10)	ASTD (4C, 70 + 10 + 20)	ASTD (3C, 80 + 10 + 10)
MC1	72.43	69.62	76.72
MC2	**73.17**	**70.23**	**78.62**
Baseline	65.58% [9]	65.05% [13]	68.60% [22]

The bottom line shows the baselines (previous highest accuracies attained) corresponding to each classification task.

**Table 14:** Accuracy with multiclass ASTD datasets, step 13 removed from preprocessing.

Models	Accuracy (%)	
	ASTD (4C, 80 + 10 + 10)	ASTD (3C, 80 + 10 + 10)
MC1	69.23	71.26
MC2	**70.32**	**74.35**

**Table 15:** Accuracy with multiclass ASTD datasets, step 20 removed from preprocessing.

Models	Accuracy (%)	
	ASTD (4C, 80 + 10 + 10)	ASTD (3C, 80 + 10 + 10)
MC1	67.65	72.69
MC2	**68.38**	**73.14**

**Table 16:** Accuracy with binary datasets ASTD and ATDFS (see text for further explanation of 86.00%).

Models	Accuracy (%)	
	ASTD (2C)	ATDFS (2C)
MC1	**90.06**	92.63
MC2	89.49	**92.96**
Baseline	85.58% [22]	86.00% [26]

**Table 17:** Accuracy with binary ASTD, step 13 removed from preprocessing.

Models	Accuracy (%)	
	ASTD (2C)	ATDFS (2C)
MC1	87.11	90.12
MC2	**88.56**	**90.86**

**Table 18:** Accuracy with binary ASTD, step 20 removed from preprocessing.

Models	Accuracy (%)	
	ASTD (2C)	ATDFS (2C)
MC1	86.19	89.23
MC2	**87.83**	**89.68**

## Data Availability

This research is based on public datasets already known to the research community.
